# Innovative Design of a Cloud Tour Guide Robot for Smart Cities under the Principle of System Innovation Design

This article has been retracted.

**DOI:** 10.1155/2022/4971849

**Published:** 2022-07-11

**Authors:** Jingjing Du, Neesa Ameera Mohamed Salim, Wan Zamani Wan Zakaria, Yanhui Gu, Jiahui Ling

**Affiliations:** ^1^College of Creative Arts, Universiti Teknologi MARA, Shah Alam, Malaysia; ^2^College of Art and Media, Suqian University, Suqian, Jiangsu, China; ^3^College of Design and Art, Huaiyin Institute of Technology, Huai'an, Jiangsu, China; ^4^Nanjing Institute of Technology, Nanjing, Jiangsu, China

## Abstract

In light of the ongoing occurrence of epidemics, the general populace frequently makes the decision to curtail their nomadic lifestyle in order to protect both their health and their safety. This has resulted in a number of issues, the most notable of which are the drop in the people's living happiness index and the poor business that the tourism industry has been experiencing as a result. Therefore, the idea of “cloud tourism” is undoubtedly the first candidate for the tourism industry, and in order to meet the requirements of cloud tourism, it is necessary to have an entirely new system to serve this, of which the scenic guide robot is an important part. At the same time, the quickening development of 5G technology offers solutions that may be put into practice for the multifurther IoT's expansion in smart cities. People will be able to experience the real outdoors without having to leave their homes, which will improve the people's well-being and alleviate the chilly status quo in the tourism industry. This is the plan, and it will be accomplished through the use of innovative guide robots that will make the experience more convenient and reliable.

## 1. Introduction

Around the time of the Chinese Spring Festival in the year 2020, an unprecedented outbreak of the COVID-19 virus occurred. The virus quickly spread across the country and even the world, which had a devastating effect on the social and economic development of China as well as the people's day-to-day lives. At this time, in response to the unexpected outbreak of the coronavirus, the entirety of the country has collaborated in an effort to combat the virus, an effort that has resulted in both gains and effects. The effect of large epidemics on the tourism business is an age-old problem that is still being investigated by scientists and technologists working in the tourism sector today. The impact of the epidemic on the tourism industry comprises not only the indirect losses produced by a large number of tourism companies and practitioners associated with the industry but also the direct losses incurred by a large number of tourism enterprises that are related to one another. Major issues that cannot be avoided and are difficult to solve by tourism experts and researchers today include the following: how to solve the challenges and practical difficulties faced by the epidemic in this critical situation; seriously analyzing and judging their impact and situation; and rationally searching for their causes and response options to the threat posed by the epidemic. By actively participating in the prevention and control of the epidemic, how to solve the challenges and practical difficulties faced by the epidemic in this critical situation; seriously analyzing and judging their impact and situation; and seriously analyzing and step-by-step, the effects of the epidemic on the travel and tourism business have become more apparent. The travel industry, which was anticipated to experience a surge during the Chinese New Year holiday, was forced to press the “pause button” due to the need to effectively prevent and control the epidemic. Prior to this, the majority of travel companies had already made their preparations and investments for the best phase of the season to welcome customers during the Chinese New Year holiday. The issue of “refund, change, and stop” orders placed with travel service providers has become increasingly apparent, with scenic spots basically maintaining zero revenue since the Chinese New Year, and with restaurants, hotels, offline leisure, and entertainment, as well as other types of business services basically shutting down, leaving travel companies in a state of passivity. For a very long time, tourism companies have had to contend with increased cost pressures, the majority of which take the form of wage payments for tourism company employees, loan repayments, initial capital investments, order refunds, interruptions to construction work, and a greater amount of pressure on tourism companies and other tourism practitioners.

On the other hand, as people's cultural living standards continue to rise, they are devoting an increasing amount of attention to the fulfillment of their spiritual requirements, which has resulted in this aspect of vacationing becoming an essential component of the whole experience. The design of the cloud tourism guide robot should take into full account the cultural ecology of each scenic area as a cornerstone. Furthermore, under the premise of meeting functionality requirements and protecting the environment, the design should then consider the aesthetics of culture and art, which will ensure that the guide system for each scenic area is one of a kind and distinctive. The display of regional cultural traits inside the scenic tour system has the potential to become a unique symbol that visitors can use to become familiar with the local culture and traditions [1, 2].

Both ground patrol robots and aerial drones have reached a high level of development in today's society, and research on various types of navigation systems has a solid foundation. As a direct result of the epidemic, there has been a significant rise in the country's utilization of online services, and the idea of “cloud services” has emerged as a major movement. Additionally, the concept of “cloud tourism” has emerged as a primary source of concern for the country's citizens. The cloud tourist guide robot has opened up new potential for economic growth as a result of its ability to more effectively cater to the requirements of locals in terms of cloud tourism.

The term “cloud tourism” refers to a tourism solution that utilizes “cloud computing” technology to establish a service integration for the entirety of the tourist process. This solution combines online and offline, virtual and real aspects of tourism. It is a new type of tourism that makes use of online virtual technology to process data from tourist destinations in complete detail, making it possible to travel the world without really having to leave your house. Guided robots are robots that guide the user through the entirety of the tourism process in the tourism system. Guided robots are also required to organize the management of nodes between attractions in the tourism area so that they can provide the user with a comprehensive and well-organized tourism experience.

The ancient Greek word synistanai, from which we get the word “system,” is composed of the words “cooperation” and “building.” The term system comes from this word. The idea of a system refers to an integrated whole that serves a certain purpose and is made up of a number of components that are related to one another and work together. The idea of a system does not shed any light on the nature of the world in and of itself. Thinking in terms of systems has been practiced and applied instinctively for a significant amount of time. It was not until the latter part of the 19th century that it was given significant consideration, enriched and developed, and utilized in a variety of different contexts. The all-encompassing view of the system is the fundamental principle underlying systems thinking. To put it another way, “look at the forest first, then focus on the individual trees.”

Analysis and reasonable screening of the properties of the guide robot and its required functions to adapt to the requirements of scenic spots and residents, using a variety of professional knowledge and technology, reasonable selection and use of materials to systematically solve the overall problem based on the innovative design concept of the system, the design is based on smart cities, combined with the needs of residents for travel under the current epidemic background, analysis, and reasonable screening of the properties of the guide robot, and its required functions to adapt to the requirements of scenic spots and residents. A management and dispatching system, as well as a remote cinematic reality system, will be provided, in addition to the design of a service robot for use at trade fairs. The robot will have both autonomous reception functions as well as a panoramic visual and voice system, which can be controlled through panoramic live interaction.

## 2. Research Status: History of the Development of Cloud Tourism Guide Robots and Bionic Robots

The highly famous wooden bull and horse from the Three Kingdoms period can be traced all the way back to the beginning of the exploration of bionic robots. In September,1960, the inaugural World Bionic Congress was held at the Ohio Air Force Base. In the decades that followed, a vast variety of bionic technologies and pieces of equipment were developed. For example, Boston Dynamics has been working on the creation of bionic robots ever since the company was established in 1992 [3, 4]. The company has made quite a name for itself by releasing a variety of robots, from the Big Dog to the Handle, which has served as a significant driving force behind the advancement of bionic robots.

### 2.1. The Concept of Cloud Tourism and Guided Robots

#### 2.1.1. Concept of Cloud Tourism

Cloud tourism is the use of “cloud computing” technology to make online and offline, virtual and real tourism solutions, forming a service integration of the whole process of tourism. Under the premise of collecting the data of tourist attractions in full detail, the use of online virtual technology processing to achieve a new tourism mode of “staying at home to travel the world.”

“Cloud tourism” as a new type of the tourism service mode, to meet the majority of consumers for some part of the requirements of tourism, many cultural tourism companies and enterprises have joined the “cloud tourism” product provider team, in this context, “cloud tourism” ushered in a rapid development. Cultural tourism enterprises must also recognize the great changes that “cloud tourism” will bring to the tourism industry, seize the opportunities of the times, launch corresponding products that meet their own characteristics, and explore market potential for the recovery of the industry in the postepidemic era.

Tourists not only need to experience through various new tourism information services and network applications based on cloud and cloud computing but also need to be able to be perceived and easily used by tourists for tourism information resources, travel agency real economy, tourism activities, travelers and other aspects of basic information, more fully enjoy personalized tourism activities, and personalized tourism customization services. It is a combination of China's modern high-tech and the modern intelligent travel management system, including introduction, shopping guide, guide, and navigation of the four basic functions [5]. This definition focuses on “cloud tourism” as a new technological approach specifically designed to enhance and improve tourism services.

Compared with traditional tourism activities, “cloud tourism” elevates tourism activities from on-site experience to “in the cloud” as an experience, breaking through the limitations of geography and time, and through the function of cloud computing, tourists can enjoy the fun of tourism anytime and anywhere through one or more terminal devices.

“Cloud tourism” is considered to be a useful attempt to adapt to the crisis of the financial recession era and to buck the trend of China's cultural and tourism industry. This creative act of taking the initiative to use the new generation of information technology to seek changes, with the tourist as the service center, is a gesture that China's tourism industry should take to transform into an era of wisdom. Supported by the mobile Internet and a wealth of digital technologies, the market for smart tourism is still full of vitality and the prospects for the “cloud economy” are unlimited.

#### 2.1.2. Concept of Guided Robot

To provide a full and well-organized tourism experience for the user, guided robots, which are robots that guide the user through the entirety of the tourism process in the tourism system, are required. This is accomplished by organizing the management of nodes between the scenic spots and the scenic spots in the tourist attractions.

5G, artificial intelligence, and other emerging technologies are reaching increasingly mature stages, creating a new strategic opportunity for industrial development to promote the development of artificial intelligence information and digital system construction in China's cultural tourism service industry [6, 7]. The “cloud exhibition,” voice virtual tour, aio, virtual reality tour, and other types of tourism information experience online and offline comprehensive dissemination and application and the service mode constantly emerge with innovation, it can be seen that the current Chinese Internet tourism context “cloud tourism” in general refers to China's network tourism users and it can use the emerging network technology means to stay at home and experience online and offline tourism information. “Cloud tourism” in general refers to the current Chinese Internet tourism context “cloud tourism.”

### 2.2. Development Status and Trend of Cloud Tourism Guidance Robots

In March 2020, according to the “implementation opinions on promoting the expansion and quality of consumption to accelerate the formation of a strong domestic market” jointly issued by the National Development and Reform Commission, the Ministry of Culture and Tourism, and other departments, the quality of cultural tourism and leisure consumption will be upgraded, and various new-generation tourism information infrastructure technologies, such as the Internet, big data, cloud computing, and artificial intelligence, will be fully utilized to enhance the level of basic services of “smart cities.”

The feeling and experience of tourism services. The new large-scale enterprise digital incubation of the tourism service industry, represented by the “cloud tourism” incubation project operation model, has become a powerful policy tool for the government to alleviate the serious impact of the avian flu outbreak and accelerate the transformation and revitalization of the tourism industry. Various large tourism agencies, attractions, and Internet service platforms are actively exploring the use of a new generation of information technology, exploring efforts to achieve deep, medium, and shallow integration with modern scientific information technology, thus constantly deriving and developing a new tourism business model and new consumer scenarios for various types of tourism. “Cloud tourism” is constantly innovating and inspiring us to tap into the huge market potential of intelligent leisure tourism in China, becoming one of the ways to optimize the structure of the tourism industry.

### 2.3. Research and Analysis of Cloud Tourism Guide Robots

In 2019, the State Council issued the “opinions on further stimulating the potential of culture and tourism consumption,” which states that we should promote the mutual integration of culture, tourism, and modern technology and develop a new generation of immersive and experiential culture and tourism consumption content based on 5G, ultra-high definition, augmented reality, virtual reality, artificial intelligence, and other technologies. With elaborate process design and advanced technology, “cloud tourism” is dedicated to providing people in front of the screen with an immersive and beautiful experience [8]. The emotional experience of being there is the “immersive” experience, which consists mainly of the human sensory and cognitive experience of oneself. Therefore, the development path of “cloud tourism” is to focus on enhancing the immersive experience of visitors from two perspectives: visual sensory and cognitive. New digital technologies, such as 3D holographic projection, ar, VR, and mr, have greatly enriched the visual and sensory experience of modern people. Many domestic and foreign companies are researching and developing service-oriented robots based on commercial applications, including Savioke, a hotel service-oriented robot that can be used to deliver disposable towels, toothpaste, and other necessities to guest rooms. When the hotel staff swipes the room number on the robot's touch screen, the Savioke will automatically arrive in the specified room. But rather than being unable to communicate with the customer, Savioke relies solely on text and images on the display to interact with the customer. The Simbe robot, used in the retail sector, can scan all the shelves of a supermarket in 30 to 40 minutes and obtain an average of 15,000 to 20,000 products per hour [9]. We also have the cobalt, an indoor security sensor machine developed by Dr. Travis Deyle, which has a built-in sensor that allows us to move people and objects around at all times and to identify all people and other objects accurately, and we can also determine whether the person has the power to detect or micro dynamically detect in the building, that is, to check whether the doors and windows in a room are open. This means that we can check whether doors and windows are open in a room and that we can report to the police any leaks or potential fire risks, or even misplacement. Domestic companies, mainly represented by Xinsong, are in the first Coworth and Silver Star intelligent education robots. They focus on modeling when designing their robots, and do not completely abandon the idea that robots should look like people, providing functions that are not rigidly required by users and lacking in functionality. At the same time, the high price of these robots is a very big obstacle on the road to their popularity.

Service robots are intelligent products for consumer-oriented robots in the future, and the demand for scenarios is the basis for the commercialization of robots, and development teams should focus more on applying robots to different scenarios to solve practical problems. Commercial autonomous mobile robots (see Figure 1) must interact effectively with other types of human technology in order to achieve seamless connectivity between robots, intelligent hardware, and application scenarios, and while robots face high technical barriers, the design of human-machine interaction interfaces for mobile machines based on psychology is also an extremely important one. It can bring considerable convenience to users in segment areas, technical specifications, and friendly interaction design in the world. In addition to household cleaning robots, there are very few typical representative works. With a focus on the exhibition service scenario, we are committed to designing a commercial service robot that is not only reliable, versatile, and has excellent interaction design but also elegant, easy to customize, and cost-effective.

### 2.4. Market Demand and Significance of Cloud Tourism Guide Robots

The design is based on the smart city, combined with the current epidemic in the context of the needs of the residents of outbound tourism, analysis, and reasonable screening to adapt to the scenic area and the residents of the properties of the guide robot and its required functions, using a variety of professional knowledge and technology, reasonable selection and use of materials to systematically solve the overall quality and structure, cruise power and energy supply, obstacle avoidance, information collection, image processing, and other issues.

#### 2.4.1. Market Demand Analysis of Cloud Tourism Guide Robots

1. From the perspective of environmental management, China is a vast country with countless tourist attractions in all regions, but the ecological protection of scenic spots has always been a top problem everywhere. The concept of cloud tourism avoids direct contact between tourists and the ecology of scenic spots, thus reducing the cost of ecological protection and intervention in the natural environment and allowing tourists to enjoy the scenery more conveniently.
2. From the perspective of humanistic care and economic recovery, in the context of the epidemic, the residents' lives are monotonous and dull when they are restricted from travelling. The cloud tourism guide robot can help the residents to enjoy the scenery remotely and “travel” without leaving home, which can not only add interest to the residents' lives during the epidemic but also increase the income of scenic spots to subsidize the losses caused by the epidemic.
3. From the psychological point of view of tourists, the tourist attraction guide system exists to achieve the guidance function for tourists. An excellent tourism guidance system can not only correctly guide users to the attractions but can also subconsciously show users the historical and cultural heritage behind the scenic spots. Generally speaking, a good tourist guidance system can enrich the sensory experience of visitors, touch their emotions, introduce them to the history and culture of the area, and increase their relevance to the area.

#### 2.4.2. Relevance of Cloud Tourism Guide Robots

*(1) Reduce the Impact of COVID-19 on the Tourism Industry*. In January 2020, the outbreak of Newcastle pneumonia swept the country in an instant. Although the government took timely preventive measures to reduce losses, it still had a serious impact on the country's economic and social development and people's lives. The impact of the epidemic on the tourism industry is divided into two parts: direct losses including tourism enterprises and their related employees, and indirect losses including tourism-related industries such as catering, accommodation, and other industries. How to deal with the crisis in the tourism industry has become a new challenge for the industry.

In recent years, there have been two major epidemics in the country, SARS in 2003 and the new crown in 2020. Prior to the start of the epidemic, as the national economy continued to develop and overall income levels gradually increased, so did the population's demand for spiritual enjoyment, such as tourism, which became one of the key elements of modern lifestyle consumption and provided new revenue opportunities for countless regions. So, with tourism booming, the blow of the new crown in 2020 will be huge [10, 11], especially in areas that rely on tourism to drive the local economy, and the new crown will undoubtedly be a fatal blow to the economy. In addition to government subsidies, the tourism industry is also looking for new opportunities to develop and explore new forms of tourism.

*(2) Protecting the Ecology of the Landscape*. As the population's demand for tourism continues to rise and tourists flock to scenic areas in large numbers, the cost of ecological conservation in scenic areas is also increasing. However, for many scenic spots, such as famous monuments and Dango landscapes, the damage caused by human activities is irreversible and malicious acts of vandalism to these spots are not uncommon. Some scenic spots must resort to restricting the number of people entering the park for the sake of the ecology of the area. In this context, cloud tourism can be a good solution to these problems, as it avoids direct contact between visitors and the attractions, and allows the area to accommodate more visitors, allowing them to enjoy the landscape more fully. The goal of the “cloud tourism” concept is a three-dimensional panorama, that is, three-dimensional projection that gives a sense of immersion. The focus of 3D projection is on data collection, and the combination of aerial drones and patrol robots allows for the most comprehensive data collection possible.

*(3) Technical Support for the Development of the New Tourism Concept of “Cloud Tourism”*. In recent years, as people's living standards improve, material satisfaction is no longer the only pursuit of life, but the satisfaction of spiritual needs has become an important part of the tourism experience, gradually giving rise to the concept of “travel without leaving home.” Therefore, the emergence of cloud tourism guide robots has made cloud tourism a reality. The design should incorporate the different cultural and ecological aspects of each scenic spot as the cornerstone of the design, and meet the principles of functionality, artistry, and ergonomics, so that the robot can not only present the cultural characteristics of the region but also provide people with the historical and cultural connotations and humanistic meanings behind these scenic spots, becoming a unique scenic spot for the public.

### 2.5. Cloud Tourism Guide Robot Classification: Ground Patrol Robots and Aerial Patrol Drones

The cloud tourism guide robot is divided into two parts: a ground patrol robot and an aerial drone, which can thus provide a more comprehensive view of the tourist scenery. Under the planning of the intelligent system, the aerial drone can follow a prescribed route for travel photography, giving visitors a bird's eye view from above. The drone is also equipped with an autonomous obstacle avoidance function. With the technical support of a small radar and infrared scanning, the drone can intelligently avoid obstacles and avoid crashing into objects. The camera installed on the drone not only collects and processes information on the scenic landscape, but also monitors the internal environment of the scenic area, and when special conditions are detected, they are uploaded to the control center via the cloud platform and handed over to the personnel responsible for handling them. Ground patrol robots and aerial drones work together under the command of the guidance system to show visitors a comprehensive view of the scenery.

## 3. Basic Concepts and Connotations of System Innovation Design

This topic is based on the system concept of the product design and system thinking to apply and explain the concept of the system, the concept of the product system and various aspects of the system concept of the product design, on the basis of the concept and connotation of system innovation design, to explain the internal and external properties of the product system, functional properties and the characteristics of the product system design in terms of wholeness, openness, extensibility, and so on.

### 3.1. Basic Concepts of the System

The word system is derived from the Greek word “synistanai,” which is made up of the roots “cooperation” and “construction.” The concept of a system is an unified whole with a specific function consisting of a number of interrelated and interacting elements.

#### 3.1.1. Background and Development of the Emergence of Systems Science

*(1) Humanity Has Gone through a Process of Understanding the World from Synthesis to Analysis to Synthesis*. Bertalanffy's general systems theory, Schenone's information theory, and Wiener's cybernetics are all theories of systems, and are known as the three major theories of the twentieth century [12]. They have been applied to scientific research, engineering design, social management, and many humanities and social sciences, and have accordingly given rise to modern design methods such as systems engineering, control engineering, and information engineering.

Systems thinking it has long been used unconsciously as a concept and a way of thinking. It was only in the second half of the 19th century that it was taken seriously, enriched and developed, and used in various ways. A system can be seen as an “ensemble of processes,” which is separated from its surroundings by boundaries and linked to them by inputs and outputs, while maintaining its own function and stability, essentially acting as a “transformation.” At the same time, the system can be divided into subsystems at various levels according to different connections, and under these subsystems there are elements. The “elements, structure, state, and process” of a system are called the “four elements” of a system.

Thus, the concept of a system does not tell us what the world itself is but how to see it.

### 3.2. The Concept of Systems Thinking

The core idea of systems thinking is the holistic concept of the system. That is, “look at the forest first, then the trees.” Systems thinking is nonmonolithic, it is bi-directional, and its logical starting point is synthesis, that is, comprehensive analysis and synthesis with feedback from each other.

Systems thinking is primarily concerned with “reductionist” thinking, which is commonly used in modern scientific research. In his book “Discourses on Method,” R. Descartes, an important representative of “reductionist” thinking, gave four principles to guide one's reasoning.

The first requires that “impatience and prejudice” be avoided and that only clear and distinct ideas be accepted.

The second requires that the problem under consideration be divided into as many parts as possible and necessary in order to obtain a clear solution.

The third requires a gradual progression from simple to the complex.

The fourth article requires complete analysis without any omission.

The second of these is considered to be the most important principle that has ruled the Western scientific method for 350 years, and has been described as “the principle of analytical reduction that has characterized the Western intellectual tradition.” It represents a one-way linear way of thinking from analysis to synthesis.

For example, the “Ding Pei Palace”-an account from the Meng Xi Pen Tao-is a famous project guided by a systematic approach.

During the reign of Emperor Zhenzong Dazhong Xiangfu, the capital city of Bianliang (now Kaifeng) was destroyed by a fire that reduced the entire palace to rubble [13]. After the disaster, Emperor Zhenzong Zhao Heng appointed the Duke of Jin - Ding Pei - as the repair envoy to preside over the restoration of the palace.

  After receiving the order, Ding Pei started his work.

1. “The Earth was far away” and he first ordered the digging of the street in front of the palace to collect the Earth. Within a few days, the street was dug into a wide ditch.
2. Then he ordered to divert Bianshui into the ditch and use “bamboo rafts and boats” to transport building materials “to the palace gate.”
3. After the restoration of the palace, the rubble and grey soil were filled into the ditch to “resume the street.”

In this way, “one move was made, and three services were performed,” “saving trillions of dollars.”

If the project is divided into three parts, the first is to transport the rubble outside the city, then to take the soil from outside the city to make tiles and bricks, and then to transport the building materials from Bianshui via land. Ding Duyi did not do all three separately but coordinated them as an organic whole, saving a great deal of human, financial, and material resources.

Therefore, the method of considering the thing under the study as a whole, seeing the connection between the elements and coordinating them from the perspective of the whole, is the method in line with systemic thinking (see Figures 2 and 3).

### 3.3. The Concept of Product Systems

#### 3.3.1. Hierarchical Nature of the Product Structure

The hierarchical nature of the system structure is an important property of the system.

The hierarchical nature of the product structure refers to the fact that due to the differences in the elements of the system and the way they are combined, the system organization shows an hierarchical order in terms of status, role, structure, and function, and a system level with qualitative differences is formed. At the same time, the systems and elements that form this level, the high-level systems, and the low-level systems are relative.

#### 3.3.2. Dual Function of the System

On the one hand, it needs to be linked to the elements in that system to form a synergistically integrated unified system.

On the other hand, it is a subsystem of a larger system, and it plays the role of an element in this larger system, forming the basis of this larger system.

#### 3.3.3. Relationships between Individuals and Sets and Species and Classes of Systems

While hierarchy reveals the hierarchical nature of systems vertically, typology reveals the multiple states of systems and their commonalities horizontally.

A type often has multiple levels, and systems at the same level can have different types.

#### 3.3.4. Three Factors of the Product System

Elements, elements and systems are a pair of relatively existing categories.

Structure is the way in which a number of elements interact with each other.

Function is the order and ability of a system to interact with its external environment.

The process of the product design is in fact a process of communication between the designer and the user, which is made up of a system by communicating with each other through the product [13]. The designer expresses his design ideas through the product to reflect the user's requirements. The success of a product lies in its ability to achieve communication between the designer and the user.

For example: the mouse. Its color, its size, the feel of its grip, the feel of its movement, the feel of the keys when they are struck, and even the sound of the keys when they are struck are all channels through which the designer communicates his message. If the message is successfully and accurately communicated and is accepted by the user, the product is a success. The user's use of the product can be fed back to the designer through various channels, which can provide a basis for the designer's next design, a cyclical process that forms a system.

## 4. Design and Implementation of the Guide Robot

### 4.1. Conceptualization of the Design of the Guided Tour Robot

#### 4.1.1. Conceptual Requirements

1. The chassis of the robot is modular, and it is equipped with anticollision mechanisms. These systems prevent the robot from rolling over at greater speeds and from tipping over when it is braking.
2. The robots have a sophisticated appearance that was intentionally created for them to utilize in industrial settings.
3. The robots are able to communicate with the platform of the management system, which then displays real-time information about all of the robots on the exhibition map. Additionally, the robots are able to send an immediate alert to the management system whenever the machine comes across an unexpected situation while it is operating, and they are able to automatically return to the charging area whenever their power supply becomes low.
4. Remote users have access to panoramic information about the venue, a feature that allows visitors who are not on-site to participate in the show at anytime and anywhere, and media workers can record or even broadcast live from the show through this device.
5. Visitors who are not on-site can participate in the show at anytime and anywhere. Monitoring of the system's security is another function that the machine provides [14–16].

### 4.2. Design Notes for the Guided Tour Robot

#### 4.2.1. Design of the Main Body Shape

The chassis is designed with an anticollision device, which increases the reliability of the robot, prevents the robot from tipping forward when braking to avoid obstacles at higher speeds, and effectively solves the phenomenon of drifting and skidding or overhanging when travelling or turning on the smoother ground of the exhibition. The whole chassis is designed in a modular way, which makes it easy to disassemble and modify or repair later and allows for some expandable sensor jacks to facilitate customization according to customer needs. The feasibility will be verified by the corresponding motion simulation software (see Figures 4 and 5).

#### 4.2.2. UAV Sections

Immersive experience devices, represented by VR glasses, have hit the market at a very low price and are starting to gain popularity. Users can use these devices to browse the panoramic impact of the robot capture, unlike the nature of VR (virtual reality) content, our system provides content that uses the audio and video data captured by the robot to reconstruct the real situation of the show in real time in three dimensions [17]. This feature allows visitors who are not on-site to participate in the show at any time, and media workers can record or even broadcast live from the show with this equipment. As well as combining drones with wheeled robots, the system transmits the surroundings to the robots in real time, providing more accurate routes for robot guidance and visual enjoyment for users at high and low altitudes (see Figures 6–9).

#### 4.2.3. Color Use and Stylistic Features

The overall white color is the main color, complemented by a low saturation, high gloss blue, which does not clash with the ambient color. The white color is simple and elegant, harmonious, and quiet. The low-saturation, low-transparency secondary colors are stylish and visually appealing.

The overall appearance of the robot is simple and generous, without too much decoration, and the overall style is rounded, but at the same time, the design of the storage space is handled with a hard element. The display is located on a rounded surface, which makes it easy to operate without losing its aesthetic appeal.

Here we give three product dimension drawings (see Figure 10).

### 4.3. Cloud Tourism Guide Robot Interaction System

#### 4.3.1. Interaction Analysis of the Cloud Tourism Guide Robot

The concept of interaction design is a way of thinking that must be followed throughout the entire process of interaction design to meet the needs and goals of the user, to achieve organic integration between the user and the design practice, and to promote interaction between the user's emotions and the designer in relation to the design concept. In the key area of architectural design, the goals and objectives of the interaction concept are to enhance the experience of designer interaction and to facilitate a strong connection between the designer and the product or the service. The goal of the visitor downloading APP is not just to act as a guide, but to give them something new to do, even if only after the online tourism campaign has officially ended, so that they cannot continue to pay new attention to it themselves, which effectively enhances the sense of interaction participation of local tourists at the same time, and can also significantly enhance the local online tourism media brand and industry awareness [18].

The simplicity of the manual mode of APP operation is very important, but of course the user is converted from the touch mode of the human-machine interface to the voice mode of operation, through a variety of operating methods, such as smartphones and a network voice, eliminating the tedious manual information input, functionality will be greatly enhanced, then the interaction experience in the tourism guide system will be very smooth [19, 20]. The deepening and strengthening of trade between China and the world have brought more and more expatriate users into China and travel to various scenic spots, but they often have a very low level of acceptance and experience of tourism because of the language barrier. Language diversity can be very effective in improving this lack of acceptance and experience.

Here, we give an interaction design of a cloud tourism guide robot (see Figure 11).

#### 4.3.2. Interaction Design of the Cloud Tourism Guide Robot

## 5. Conclusion

This topic explores a new “cloud tourism” guide robot solution, through the shape and structure of the guide robot design, and then by the APP interactive system for process optimization, to achieve the “cloud tourism” goal. This was accomplished after extensive discussion and research, combined with the production of 3D-aided technology. The concept of a brand-new kind of the “cloud tourism” guide robot serves as the foundation for this project. In addition, the design is based on the multi-IoT in smart cities, which makes it simpler to cross borders from one city to another and makes the solution simple to learn and efficient. This results in a more realistic way of experiencing cloud tourism and gives people the opportunity to experience the outdoors without having to leave their homes. After the completion of the entire system, based on the actual operation effect, the guide robot solution has a more practical application value, has a broad development prospect in the future consumer market, and has the potential to become the mainstream of the social tourism mode. These are all claims that are supported by the fact that the solution has been put into operation.

## Figures and Tables

**Figure 1:** Autonomous mobile robots are developed by companies based on commercial application scenarios.

**Figure 2:** Portrait of Ding Paixiu palace (tencent).

**Figure 3:** The site of Ding Wei's palace restoration (tencent).

**Figure 4:** Conceptual sketch design.

**Figure 5:** Program defined design.

**Figure 6:** Introduction and description of the structure section.

**Figure 7:** Electronic screen display.

**Figure 8:** Partial rendering of the storage structure.

**Figure 9:** Structural rendering of components.

**Figure 10:** Product dimensional drawing. (a) Top view. (b) Side view. (c) Front view.

**Figure 11:** APP interaction interface design. (a) Main interface design. (b) Opening interface design. (c) Main menu design.

## Data Availability

The dataset used to support the findings of this study are available from the corresponding author upon request.

## References

[1] Hatchuel A., Weil B. A new approach of innovative design: an introduction to CK theory.

[2] Kawaguchi D., Nakamura R., Hadama H. Evaluation on a drone classification method using UWB radar image recognition with deep learning.

[3] Jain N., Gupta A. K., Mathur P. Autonomous drone using ROS for surveillance and 3D mapping using satellite map.

[4] Wang S., Christensen H. I. Tritonbot: first lessons learned from deployment of a long-term autonomy tour guide robot.

[5] Vasquez B. P. E. A., Gonzalez R., Matia F., Puente P. D. L. (2018). Sensor fusion for tour-guide robot localization. *IEEE Access*.

[6] Wang S., Liu X., Zhao J., Christensen H. I. Rorg: service robot software management with linux containers.

[7] Chella A., Macaluso I. (2009). The perception loop in CiceRobot, a museum guide robot. *Neurocomputing*.

[8] Matsumoto K., Imai M. Quasi-zenith satellite system-based tour guide robot at a theme park.

[9] Dong H., Zhang X., Kong D., Zhang B. Design and implementation of intelligent tour guide system in large scenic area based on fog computing.

[10] Tsai H. Y., Kuwahara Y., leiri R., Hishiyama R. (2019). Vision-based indoor positioning (VBIP) - an indoor AR navigation system with a virtual tour guide. *Collaboration Technologies and Social Computing*.

[11] Biswas J., Veloso M. (2013). *Multi-sensor mobile Robot Localization for Diverse Environments*.

[12] Dellaert F., Burgard W., Fox D., Thrun S. Using the condensation algorithm for robust, vision-based mobile robot localization.

[13] Saffiotti A., Broxvall M. PEIS ecologies: ambient intelligence meets autonomous robotics.

[14] Moon S. W., Kim Y. J., Myeong H. J., Kim C. S., Cha N. J., Kim D. H. Implementation of smartphone environment remote control and monitoring system for Android operating system-based robot platform.

[15] Hnatiuc M., Paun M., Dussart J. Path recognition using mobile phone.

[16] Iida M., Suguri M., Uchida R. (2013). Advanced harvesting system by using a combine robot. *IFAC Proceedings*.

[17] Gopal L., Loong A. W. W. Designing and implementing a wi-fi enabled mobile robot.

[18] Batty M., Axhausen K. W., Giannotti F. Smart cities of the future. *The European Physical Journal - Special Topics*.

[19] Chourabi H., Nam T., Walker S., Garcia R. G., Mellouli S., Nahon K. Understanding smart cities: an integrative framework.

[20] Geels F. W. (2004). Understanding system innovations: conceptual synthesis. *System innovation and the transition to sustainability: Theory, evidence and policy*.

